The article "Perivascular radiofrequency renal denervation lowers blood pressure and ameliorates cardiorenal fibrosis in spontaneously hypertensive rats" was published in 2017. Journal: PLoS One.

# Perivascular radiofrequency renal denervation lowers blood pressure and ameliorates cardiorenal fibrosis in spontaneously hypertensive rats

**DOI:** 10.1371/journal.pone.0176888

**Published:** 2017-04-28

**Authors:** Shujie Wei, Dan Li, Yan Zhang, Linan Su, Yunrong Zhang, Qiang Wang, Dachun Yang, De Li, Yongjian Yang, Shuangtao Ma

**Affiliations:** 1 Department of Cardiology, Chengdu Military General Hospital, Chengdu, Sichuan, China; 2 Department of Internal Medicine, Shapingba People's Hospital, Chongqing, China; University Medical Center Utrecht, NETHERLANDS

## Abstract

**Background:**

Catheter-based renal denervation (RDN) is a promising approach to treat hypertension, but innervation patterns limit the response to endovascular RDN and the post-procedural renal artery narrowing or stenosis questions the endovascular ablation strategy. This study was performed to investigate the anti-hypertensive and target organ protective effects of perivascular RDN in spontaneously hypertensive rats (SHR).

**Methods:**

SHR and normotensive Wistar-Kyoto (WKY) rats were divided into sham group (n = 10), radiofrequency ablation group (n = 20) in which rats received bilateral perivascular ablation with radiofrequency energy (2 watts), and chemical (10% phenol in 95% ethanol) ablation group (n = 12). The tail-cuff blood pressure was measured before the ablation and on day 14 and day 28 after the procedure. The plasma levels of creatinine, urea nitrogen, and catecholamines, urinary excretion of electrolytes and protein, and myocardial and glomerular fibrosis were analyzed and compared among the groups on day 28 after the procedure.

**Results:**

We identified that 2-watt is the optimal radiofrequency power for perivascular RDN in rats. Perivascular radiofrequency and chemical ablation achieved roughly comparable blood pressure reduction in SHR but not in WKY on day 14 and day 28 following the procedure. Radiofrequency-mediated ablation substantially destroyed the renal nerves surrounding the renal arteries of both SHR and WKY without damaging the renal arteries and diminished the expression of tyrosine hydroxylase, the enzyme marker for postganglionic sympathetic nerves. Additionally, perivascular radiofrequency ablation also decreased the plasma catecholamines of SHR. Interestingly, both radiofrequency and chemical ablation decreased the myocardial and glomerular fibrosis of SHR, while neither increased the plasma creatinine and blood urea nitrogen nor affected the urinary excretion of electrolytes and protein when compared to sham group.

**Conclusions:**

Radiofrequency-mediated perivascular RDN may become a feasible procedure against hypertension, and provide similar anti-hypertensive and target organ protective effects as does the chemical ablation.

## Introduction

Catheter-based endovascular renal denervation (RDN) is a promising strategy for the treatment of resistant hypertension [1–5]. The RDN not only lowers blood pressure (BP) but also plays a potential therapeutic role in sympathetic overactivity-linked disorders, including left ventricular hypertrophy, heart failure, tachyarrhythmia, insulin resistance, and chronic kidney disease [6–11]. Although the SYMPLICITY HTN-3 [12], a randomized prospective blind clinical trial, failed to show benefits from RDN for patients with resistant hypertension as compared with a sham group, the RDN is not yet dead [13, 14]. Instead, this trial promotes the comprehensive mechanistic study on the effect of RDN in the treatment of hypertension. There are several possible reasons explaining why the BP reduction in SYMPLICITY HTN-3 trial did not meet statistical significance. Tzafriri et al. evaluated benefits of endovascular radiofrequency ablation in different types of renal neural network anatomy through investigating the nerve and ganglia distribution surrounding the renal artery [15]. It demonstrated that innervation patterns may limit the response to endovascular ablation. This finding encouraged us to investigate the feasibility and effect of perivascular ablation.

Although the RDN is a relatively safe procedure, there are also complications such as renal artery stenosis which may be responsible for the recurrence of hypertension following the successful ablation. Along with the wide application of RDN, more attention has been paid to RDN-associated renal artery stenosis[16–22]. Despite of the low incidence of post-ablation stenosis, the nonsignificant renal artery narrowing and worsening of pre-existing stenosis still need to be considered. For example, the EnligHTN I trial reported that 2 of 46 (4.3%) patients showed progression of a antecedent renal artery stenosis [23]. The development of renal artery narrowing or stenosis is speculatively due to the injury of vascular endothelium during the endovascular radiofrequency ablation. In this case, the perivascular ablation could reduce or even avoid the endothelial injury and the subsequent renal artery narrowing or stenosis. Moreover, the perivascular ablation could be also an alternative for patients with stenotic or stented renal arteries.

In this study, we tested the efficacy and safety of perivascular radiofrequency ablation of renal artery in spontaneously hypertensive rats (SHR) and normotensive Wistar-Kyoto (WKY) rats. We optimized the radiofrequency ablation energy and also compared the anti-hypertensive effects of radiofrequency ablation with the chemical denervation with phenol-ethanol.

## Materials and methods

### Ethics statement

This study was carried out in strict accordance with the recommendations in the Guide for the Care and Use of Laboratory Animals of the National Institutes of Health. The protocol was approved by the Ethics Committee and the Institutional Animal Care and Use Committee of Chengdu Military General Hospital. All procedures were performed under anesthesia, and all efforts were made to minimize suffering.

### Animals

Male SHR and WKY, 8 weeks of age, were purchased from Vital River Laboratories (Beijing, China). All rats were housed in our animal facility with a 12-hour light/dark cycle and were given standard chow and drinking water *ad libitum*.

### Experimental protocol

SHR and WKY were divided into three groups: sham group (n = 10), bilateral perivascular radiofrequency ablation group (RFA, n = 20), and phenol-ethanol ablation group (PEA, n = 12). The BP and heart rate were measured, the blood samples were collected from nicking the tail vein, and the 24-hour urine samples were collected using the metabolic cage the day before the procedure and on day 14 and day 28 after the procedure. On day 14 after the ablation, 10 rats from RFA group and 6 from PEA group were sacrificed, and the left rats in these two groups and the rats in sham group were sacrificed on day 28 following the procedure. For the terminal procedure, rats were deeply anesthetized with sodium pentobarbital (100 mg/kg, i.p.) and intracardially perfused with 0.9% saline solution. Then, the heart, kidney, and renal arteries were harvested for histological analysis.

### Perivascular RDN

Rats were anesthetized with sodium pentobarbital (50 mg/kg; i.p.) and given a dose of ketoprofen (16 mg/kg; s.c.) for pain relief. The abdominal area was shaved and scrubbed with a 7.5% povidone-iodine solution. An incision was made in the midline. Renal arteries and veins were identified and exposed. For the radiofrequency ablation, a 5Fr ablation catheter (APT Medical Inc., Shenzhen, China) was placed on the renal artery. A dispersive electro-conductive plate was put on the shaved back of rats as a reference electrode. Two upper and two lower points on each renal artery were chosen for ablation. The optimized radiofrequency energy was set to 2 watts after trying with 1, 2, 3, and 4 watts (n = 3 WKY rats for each group). Radiofrequency energy was applied to each point (Fig 1A) and lasted up to 60s. The temperature of tissue-electrode interface was maintained to 40°C during the procedure. For chemical ablation, the denervation was performed by gently painting the renal artery with 10% phenol in 95% ethanol solution as described in the previous report [24]. As a sham operation, renal arteries were exposed but neither radiofrequency energy nor chemical was delivered. Immediately after surgery, rats were placed in their cages that were placed on warm pads until the animals fully recovered and were moving in the cage. Rats were monitored by daily visual examination of the incision and overall condition during the first 5 days after the procedure and no adverse events were found in our experiments.

**Fig 1:** Radiofrequency-mediated perivascular renal denervation in rats. (A) a representative procedure photo. Red arrow, renal artery; black arrow, ablation catheter. (B-F) Hematoxylin & eosin-stained sections of WKY rat renal arteries after perivascular ablation with the radiofrequency power of 0- (B), 1- (C), 2- (D), 3- (E), and 4-watt (F) show that renal nerve bundles were disrupted by radiofrequency ablation with 2-, 3-, or 4-watt and that renal arteries got damaged and thinned after ablation with 3 or 4 watts. Black arrows, perivascular nerves; red arrows, damaged renal artery. Scale bar, 200 μm.

### BP measurement

Indirect systolic and diastolic BP and heart rate measurements were performed in conscious, restrained rats by tail-cuff plethysmography (BP-2010A, Softron Biotechnology, Beijing, China) [25].

### Blood and urine tests

The blood urea nitrogen (BUN) and serum creatinine (Scr) were determined by a chemiluminescence method. The 24-hour urinary excretions of potassium, sodium, chloride, and protein were also measured by a chemiluminescence method. The plasma dopamine, epinephrine, and norepinephrine were detected with enzyme-linked immunosorbent assay (ELISA) kits (AK0014NOV06007, AK0014NOV06008, AK0014NOV06006, Elabscience, Wuhan, China).

### Histology

The rat heart, kidneys, and left renal artery were fixed with 4% paraformaldehyde, dehydrated, embedded in paraffin, sliced in 5μm-thick slides, and stained with hematoxylin & eosin, Masson trichrome, and Movat pentachrome stains and analyzed under the Olympus BX41 microscope (Olympus Corp., Tokyo, Japan) [26]. The percentage of the fibrous area was calculated by ImageJ software.

### Immunohistochemistry

Right renal arteries with perivascular tissues were cut into three segments: proximal (close to aorta), middle, and distal (close to kidney). The arterial segments were fixed, embedded in paraffin, and cut into sections of 5μm in length. Every 5^th^ section was collected and 20 sections from each segment were stained with immunohistochemistry for tyrosine hydroxylase (TH). Therefore, 60 sections from each rat were analyzed. The immunohistochemistry staining for TH was performed using rabbit anti-TH antibody (dilution: 1:200, ab41528, Abcam, Cambridge, UK) [27]. After being washed, sections were incubated with goat anti-rabbit immunoglobulin G biotinylated secondary antibody (dilution: 1:200; SA1022, Boster, Wuhan, China) for 1 h at room temperature, and then detected using a DAB kit (AR1000, Boster, Wuhan, China). Sections were examined with an Olympus BX41 microscope (Olympus Corp., Tokyo, Japan). The TH-positive area (brown) and the entire area of the sympathetic nerves in each section were measured using ImageJ software and used to calculate the percentage of TH-positive area out of the entire sympathetic nerve area.

### Statistical analyses

Continuous data are presented as mean ± standard error (SE). Comparisons between groups and among different time points were determined by two-way ANOVA with Bonferroni *post-hoc* tests (SPSS Inc., Chicago, IL, USA). Probabilities of P<0.05 were considered statistically significant.

## Results

### Perivascular radiofrequency ablation-mediated RDN

Radiofrequency energy set at 1 watt to 4 watts was applied to the WKY rat renal arteries (Fig 1A), and 0 watt was used as control (Fig 1B). From the histology of the ablated arteries, the perivascular nerve was not significantly damaged by ablation with 1 watt, while was substantially destroyed as axon disruption or loss by ablation with 2, 3, or 4 watts (Fig 1C–1F). However, radiofrequency energy at 3 and 4 watts caused damage to renal arterial wall, displaying thinner than normal vascular wall (Fig 1E and 1F). Therefore, 2-watt was chosen for the further experiments.

### Perivascular RDN lowers BP

On day 14 and 28 after the procedure, both systolic and diastolic BP of SHR in either RFA or PEA group was significantly reduced when compared to sham group (Fig 2A and 2B). Systolic BP of SHR in RFA group was lower than that in PEA group on day 14, but was similar between RFA and PEA groups on day 28 (Fig 2A). Diastolic BP of SHR in RFA group was similar to that in PEA group on day 14, but was higher than PEA group on day 28 (Fig 2B). In contrast, neither radiofrequency nor chemical ablation affected the BP of normotensive WKY rats (Fig 2A and 2B). Heart rate of both SHR and WKY was significantly decreased on day 14 after radiofrequency ablation when compared to sham group but recovered on day 28, whereas the phenol-ethanol ablation didn’t influence the heart rate of both rat strains (Fig 2C).

**Fig 2:** Blood pressure and heart rate after perivascular renal denervation. The systolic (A) and diastolic (B) blood pressure (BP) and heart rate (C) of spontaneously hypertensive rats (SHR) and Wistar-Kyoto (WKY) rats the day before radiofrequency ablation (RFA) or phenol-ethanol ablation (PEA) and on day 14 and 28 after the procedure. Data are mean ± SE (n = 10 in sham group and RFA group, n = 6 in PEA group at each time point) **P<0.01 vs. the same rat strain in sham group at the same time point. ^#^P<0.05 vs. SHR in PEA group at the same time point. bpm, beat per minute.

### Perivascular radiofrequency ablation destroys renal nerves and decreases sympathetic activity

Perivascular radiofrequency ablation caused obvious injury to nerves surrounding the renal artery in both SHR and WKY (Fig 3A). Moreover, the immunohistochemical staining confirmed the damage of perivascular nerve. The sham group showed almost intact sympathetic nerves, but TH-positive area was significantly decreased in ablation groups compared to sham group (Fig 3B and 3C). Plasma dopamine, epinephrine, and norepinephrine of SHR in RFA and PEA groups were remarkably decreased on day 14 and 28 after the procedure when compared to sham group (Fig 4A–4C). In WKY rats, only plasma dopamine, but not epinephrine and norepinephrine, was decreased at these two time-points following the ablation (Fig 4A–4C).

**Fig 3:** Perivascular radiofrequency ablation destroys renal nerves. Hematoxylin & eosin-stained (A) and immunohistochemistry (anti-tyrosine hydroxylase (TH) antibody)-stained (B) sections of rat renal arteries of spontaneously hypertensive rats (SHR) and Wistar-Kyoto (WKY) rats sacrificed on day 14 after radiofrequency ablation (RFA) and on day 28 after sham procedure or RFA show that the renal nerve bundles were disrupted and the TH expression was diminished in RFA group compared to sham group. Arrows indicate perivascular nerves. (C) The percentage of TH-positive area in the entire sympathetic nerve area. Data are mean ± SE from 10 rats in each group at each time point. **P<0.01 vs. sham groups.

**Fig 4:** Perivascular radiofrequency ablation decreases plasma catecholamines. The plasma dopamine (A), epinephrine (B), and norepinephrine (C) of spontaneously hypertensive rats (SHR) and Wistar-Kyoto (WKY) rats the day before radiofrequency ablation (RFA) and day 14 and day 28 after the ablation. Data are mean ± SE from 10 rats in each group at each time point. **P<0.01 vs. sham groups.

### Perivascular RDN ameliorates cardiorenal fibrosis

Compared to WKY, SHR showed obvious cardiac fibrosis, which was attenuated in both RFA and PEA groups at 28 days after the procedure (Fig 5A and 5C). Similarly, the glomerular fibrosis in SHR was also attenuated by RFA or PEA (Fig 5B and 5D). Additionally, rat renal arteries were not damaged by perivascular RDN (Fig 6).

**Fig 5:** Perivascular ablation attenuates cardiorenal fibrosis. Masson trichrome-stained sections of heart (A) and kidney (B) of spontaneously hypertensive rats (SHR) and Wistar-Kyoto (WKY) rats sacrificed on day 28 following sham procedure, radiofrequency ablation (RFA), or phenol-ethanol ablation (PEA). The quantification of fibrous area in heart (C) and kidney (D). Data are mean ± SE (n = 10 for sham and RFA groups and n = 6 for PEA group). **P<0.01 vs. sham groups.

**Fig 6:** Renal artery after perivascular ablation. Movat pentachrome-stained sections of renal arteries of spontaneously hypertensive rats (SHR) and Wistar-Kyoto (WKY) rats sacrificed on day 28 following sham procedure, radiofrequency ablation (RFA), or phenol-ethanol ablation (PEA).

### Effects of perivascular RDN on renal function

The serum creatinine level of both SHR and WKY in RFA group was decreased when compared with sham group, while the level in PEA group is similar to sham group (Fig 7A). The BUN (Fig 7B) and the urinary excretion of potassium (Fig 7C), sodium (Fig 7D), chloride (Fig 7E), and protein (Fig 7F) were not significantly changed by RFA or PEA in both SHR and WKY.

**Fig 7:** Renal function and urinary excretions after perivascular ablation. The serum creatinine (A), blood urea nitrogen (BUN) (B), and urinary excretions of potassium (C), sodium (D), chloride (E), and protein (F) of spontaneously hypertensive rats (SHR) and Wistar-Kyoto (WKY) rats at 28 days after sham procedure, radiofrequency ablation (RFA), or phenol-ethanol ablation (PEA). Data are mean ± SE (n = 10 for sham and RFA groups and n = 6 for PEA group). **P<0.01 vs. sham group.

## Discussion

In this study, we found that perivascular radiofrequency ablation substantially destroyed the renal nerves, significantly lowered the BP, and attenuated the cardiorenal fibrosis of hypertensive rats. Additionally, these anti-hypertensive and anti-fibrotic effects were roughly comparable with the chemical ablation. Moreover, the perivascular RDN neither damaged the renal arteries nor caused renal dysfunction. These findings indicate the radiofrequency energy-mediated perivascular RDN is an effective and safe anti-hypertensive procedure for the rat model.

The endovascular ablation has a couple of limitations. Firstly, renal nerves that are far from the lumen of renal arteries are difficult to be ablated by transluminal catheter [15]. Secondly, the endothelial cell injury caused by the endovascular ablation could result in the subsequent renal artery narrowing or restenosis and worsen pre-existing renal artery stenosis [28]. The perivascular ablation procedure may be a potential strategy to overcome the above pitfalls. There are several published studies that investigated the effects of perivascular chemical RDN on BP reduction and target organ protection in rat [24, 29]. Recently, the efficacy and safety of chemical (ethanol)-mediated perivascular RDN has been tested in preclinical pig model [30], and eventually validated in patients with refractory hypertension [31]. Additionally, the feasibility of radiofrequency-mediated perivascular RDN has recently been tested in rat model [32, 33]. The present study directly compared the anti-hypertensive effects of perivascular radiofrequency and chemical ablation and found that both procedures achieved comparable reduction of BP and anti-fibrotic effects. Moreover, the present study also provided the evidence of target organ protection by perivascular RDN, which was not investigated in previous studies [32, 33]. The temporal fall in heart rate of SHR may be due to decreased sympathetic activity. Urinary sodium excretion is positively while potassium inversely associated with BP level [34]. However, urinary electrolyte excretion has no significant difference among the groups, indicating this is not responsible for the RDN-induced BP reduction. One limitation is that we didn’t correct the urinary excretion with food and drink intake. Nevertheless, our study suggests that the perivascular radiofrequency ablation is a promising alternative approach to perform catheter-based renal denervation, especially for the pre-existing stenotic and stented renal arteries.

The SHR is a well-established animal model of hypertension, which has been broadly used in the test of novel anti-hypertensive agents [35]. This strain not only displays high BP but also has target organ damage, such as myocardial and glomerular fibrosis. Moreover, the normotensive WKY rat serves as a good control for the SHR in the translational experiments. One limitation in the current study is that the SHR is not a real model of resistant hypertension. Although we validated the feasibility, efficacy, and safety of radiofrequency-mediated perirenal RDN in hypertensive rat model, a large animal model is still necessary to be used to test this procedure before it goes to clinical study. Previously, we reported a spontaneously hypertensive mini-pig model that responds well to catheter-based transluminal RDN [27]. Therefore, this hypertensive mini-pig should also be a good translational model for testing the perivascular RDN in the future. The perivascular ablation may require a bit more invasive strategy than endovascular intervention. However, the minimally invasive retroperitoneal endoscopic technology has been largely advanced. We believe the mini-invasive retroperitoneal laparoscopy would be helpful when the perivascular ablation is translated to clinical trial or practice.

The radiofrequency energy should be carefully tested and determined before the procedure. As shown in our study, high power could destroy renal arteries while low energy was not sufficient to damage perivascular nerves. A major difference between endovascular and perivascular ablation is that the target temperature in perivascular ablation should be achieved at relatively lower energy than typically seen on the endovascular catheter because of the absence of convective cooling of the ablation electrode by the bloodstream. Meanwhile, an advantage is that we can easily test the optimal energy *ex vivo* and that should be very similar to the one needed *in vivo*. In summary, the radiofrequency-mediated perivascular RDN is worth to be tested in large translational animal models.
